# Enterprise Operating State Evaluation Based on Association Rule Algorithm and Data Set

**DOI:** 10.1155/2022/1300068

**Published:** 2022-09-22

**Authors:** Shoubo Li, Haiyan Zhu

**Affiliations:** ^1^School of Management, Wuzhou University, Wuzhou, Guangxi 543002, China; ^2^School of Business, Wuzhou University, Wuzhou, Guangxi 543002, China

## Abstract

In order to further improve the evaluation quality of enterprise operating efficiency, reduce the error items and invalid items of partition, and improve the objectivity of operating condition evaluation, this study takes listed enterprises as an example and proposes an evaluation method of operating efficiency based on association rule algorithm and data set. In this method, the results of operating efficiency are scientifically analyzed from horizontal and vertical dimensions. The operating cost of total assets of listed companies is taken as indicators, and the correlation test is carried out by Kendall's tau_b. From the longitudinal comparison results, it can be seen that only 12 of the 19 enterprises in the study have small-scale changes and increase year by year, accounting for 63.16%. At the same time, there are also 6 enterprises with an overall trend of decline, which objectively reflects the reasonable operation status and operation scale of enterprises in the study.

## 1. Introduction

With the advent of the information age and the development of big data technology, the traditional economic structure, and social-economic system have undergone great changes to a large extent. For enterprises, the traditional management mode is not suitable for the current development of nature. Modern enterprise management mode is increasingly dependent on information science and technology, and the innovation and reform of enterprise management mode also promote its own development [1]. Facing the change in internal and external environment and the adjustment of market patterns, enterprises begin to attach importance to the application of various management systems, and the use of these applications also generates huge data, which is usually stored in the database, as shown in Figure 1 [2]. How to use data mining and data set analysis to deeply mine the valuable information in these data and give full play to the role of data is the focus of this research.

First of all, the connotation of enterprise operating efficiency researchis discussed. Du discussed the connotation of enterprise operating efficiency from multiple perspectives, and then discussed the source and relationship of enterprise operating efficiency. They believed that enterprise operating efficiency reflects the realization degree of enterprise operating goals, and is the comprehensive embodiment of internal efficiency and external efficiency [3]; In view of the lack of clear distinction between efficiency and benefit in existing studies, Wang et al. clarified the connotation of business efficiency and standardized terms from the theoretical and academic level, providing reference for the standardization of relevant studies [4]; Gong et al., in view of the fact that the comprehensive management efficiency of enterprises is low, after determining the basic connotation of enterprise management efficiency, combining the international advanced theory and practice, from the perspective of enterprise resource utilization and capacity improvement, combined with the concept of continuous improvement and KPI management, this paper analyzes the business process of enterprises and summarizes the KPI efficiency evaluation methods based on resources and capabilities of enterprises [5]. Second, in different enterprises operating efficiency evaluation methods, Balabanis and Stathopoulou reviewed the research status of efficiency evaluation of knowledge-based enterprises. They are based on the core characteristics of knowledge-based enterprises and the evaluation standard of MAKE. The paper puts forward the nonfinancial efficiency evaluation index system of knowledge-based enterprises from the aspects of innovation ability, human resource management ability, marketing ability, etc. It includes five indicators and 22 secondary indicators, and uses the analytic hierarchy process (AHP) to determine the weight of the evaluation system and the comprehensive index model [6]; Fachrudin et al. in the framework of the balanced scorecard, points out that the current efficiency of retail enterprise management should not only focus on financial reporting data and results, but should pay more attention to the details of the management and the use of the nonfinancial indicators, from the four dimensions of balanced scorecard, the combination of financial and nonfinancial indicators, retail enterprise management in the balanced scorecard to explore the specific dimensions of vulnerabilities, and more targeted promotion of retail enterprise performance management [7]. On the basis of analyzing the financial performance evaluation of colleges and universities, Nikolchuk established comprehensive evaluation indexes from five aspects, and took a certain college as an example to conduct the comprehensive evaluation by using the analytic hierarchy process [8]; Zhang et al. used DEA method to analyze the innovation efficiency of 11 listed logistics enterprises in 2017 and 2019, and found that some enterprises were not at the forefront of production in 2017 and 2018, and their efficiency needed to be improved. But in 2019, the efficiency was optimized and DEA effectiveness was realized. Some enterprises were more efficient in 2017 and 2018, but some problems occurred in 2019 and their efficiency decreased [9]; Duan et al. conducted a quantitative analysis and evaluation of the efficiency of 79 Chinese enterprise group finance companies in 2019 by the DEA method. The research results show that the overall efficiency of Chinese finance companies is relatively low, and the efficiency of finance companies is less affected by scale efficiency than by pure technical efficiency. In terms of industry classification, the efficiency of finance companies in petrochemical, steel, and nonferrous metals industries is better than that in other industries [10]; Based on the current situation of the bank window business and the market's expectation of the bank's due service, Cai analyzed its influencing factors and explained the structural model through analytic Hierarchy Process (AHP), quantitatively analyzed and verified the improved situation, so as to realize the process of bank's digital transformation. They combine the evaluation of the service efficiency of the electronic channel, and then analyze whether the physical resource allocation is reasonable, whether the practice of reducing the operating cost destroys the residents' demand for the basic service of the bank, and so on [11].

## 2. Association Rule Algorithm Based on Data Analysis

### 2.1. Association Rule Algorithm Based on Data Similarity

The experts with the same recommendation conclusion in the recommendation expert set *E*_*c*_ are merged into a recommendation expert group, which is defined as follows: The recommendation expert group GROUP_*i* is any subset of *E*_*c*_, namely,

(1) $$\begin{array}{c} GROUP\_E_{i}=\left\{\begin{array}{c} \left(P_{i,1},GP_{i,1}\right)⟶\left(B_{i,1},GB_{i,1}\right),\ldots ,\left(P_{i,j},GP_{i,j}\right)⟶\\ \left(B_{i,j},GB_{i,j}\right),\ldots ,\left(P_{i,m},GP_{i,m}\right)⟶\left(B_{i,m},GB_{i,m}\right) \end{array}\right\}\text{.} \end{array}$$

(*P*_*i*,*j*_, *GP*_*i*,*j*_)⟶(*B*_*i*,*j*_, *GB*_*i*,*j*_) is GROUP_*E*_*i*_'s *j* th expert, *m* is GROUP_*E*_*i*_'s elements' number, GROUP_*E*_*i*_ is a group of experts, if it satisfies the following equation:

(2) $$\begin{array}{c} B_{i,1}===B_{i,m}. \end{array}$$

The same conclusions are recommended.

The behavioral similarity between the antecedent and target customer *P*_*i*_ of the *j*th expert in the expert group GROUP_*E*_*i*_ is defined as follows:

(3) $$\begin{array}{c} Sim\left(P_{i,j},P_{i}\right)=\left|P_{i,j}\cap P_{i}\right|. \end{array}$$

After normalization,

(4) $$\begin{array}{c} {BeSim}_{j}=\frac{Sim\left(P_{i,j},P_{i}\right)}{\overset{m}{\underset{j=1}{\sum }}\left(P_{i,j},P_{i}\right)}. \end{array}$$

The weight of the *j* th expert in the expert group GROUP_*E*_*i*_ is expressed as:

(5) $$\begin{array}{c} w_{j}=\frac{\alpha \times {BeSim}_{j}+\beta \times {BeSim}_{j}}{\overset{n}{\underset{j=1}{\sum }}\left(\alpha \times {BeSim}_{j}+\beta \times {BeSim}_{j}\right)}, \end{array}$$

*m* is the number of experts in the expert group GROUP_*E*_*i*_, *α*+*β*=1 and *α*, *β* reflect the relative importance of behavioral similarity and scoring similarity in measuring the weight of experts, which can be set according to actual needs [12].

The total score of the expert group GROUP_*E*_*i*_ on the recommendation, the conclusion is expressed as follows:

(6) $$\begin{array}{c} E_{i}=\overset{m}{\underset{j}{\sum }}w_{j}\times GB_{i,j}\times f_{j}\times {sup}_{j}. \end{array}$$

According to the above algorithm steps, firstly, mining recommendation rules; Then the score value of the recommendation rule was calculated. Then the recommendation expert group was generated and the recommendations of experts in each group were assembled [13]. Finally, select corresponding expert groups according to the number of recommended items required by the system. Select the expert group with the highest total score among the selected expert groups, and its recommendation conclusion is the final recommendation result.

### 2.2. Serial Association Rule Data Set Optimization Algorithm

In view of the large time and space complexity of Eclat algorithm, changing the storage structure can achieve the purpose of reducing the size of the item set, reducing the number of intersection and shortening the escape time, etc., and the pruning strategy can reduce irrelevant item set operations, optimize the execution process, and improve the overall computational efficiency of the algorithm [14].

Let the transaction database can be shown as

(7) $$\begin{array}{c} D=\left\{T_{1},T_{2},T_{3},\ldots ,T_{n}\right\}. \end{array}$$

*T*_*n*_ is a transaction record in the transaction database, which is a collection composed of each item *T*_*n*_ with a unique identifier, namely transaction identifier (TID) [15]. Let the item set be as follows:

(8) $$\begin{array}{c} I=\left\{i_{1},i_{2},i_{3},\ldots ,i_{k}\right\}. \end{array}$$

In the above formula, *i*_*k*_ is an Item in the transaction database, usually called data Item. The collection of items is usually called Item set. The length *k* of Item set refers to the number of items contained in an Item set, and the Item set with length is called K-item set [16].

Support degree: given a global item set *I* and transaction database *D*, the support of an item set *I*_1_⊆*I* on is the percentage of transaction records *D* containing *I*. see (9), |*∗*| represents ∗'s number of collections.

(9) $$\begin{array}{c} Support\left(I_{1}\right)=\frac{\left|\left\{\left.T_{i}\right|I_{1}\subseteq T_{i},T_{i}\in D\right\}\right|}{\left|D\right|}. \end{array}$$

Confidence coefficient: given a global item set *I* and a transactional database *D*, for. two items or item sets *X*, *Y*. Among them, *X*⊆*I*, *Y*⊆*I* and *X*∩*Y*=*φ*, *A*⟶*B*'s confidence represents the ratio of the number of transaction records contained *A* and *B* in the transaction database *D* to the number of transaction records *A* contained in the transaction database *D*, as shown in

(10) $$\begin{array}{c} Confi\;de\;nce\left(X⟶Y\right)=P\left(\left.X\right|Y\right)=\frac{Support\left(X\cup Y\right)}{Support\left(X\right)}\text{.} \end{array}$$

Frequent item set: given the global item set *I* and transaction database *D*, and set the minimum support threshold Min_Sup, for any nonempty subset *I*_*i*_ of *I*, if its support satisfies formula (11) and is greater than or equal to the minimum support, *I*_*i*_ is called frequent item set.

(11) $$\begin{array}{c} Support\left(I_{i}\right)\geq \underset{10}{\mathrm{Min}\_Sup}\text{.} \end{array}$$

Strong association rule: for two projects or sets of projects *X*, *Y*, among them *X*⊆*I*, *Y*⊆*I* and *X*∩*Y*=*φ*, set association rules *X*⟶*Y*, and set the minimum support threshold Min_Sup, set minimum confidence threshold as Min_Conf, if its support satisfies formula (12) is greater than or equal to the minimum support, and its confidence satisfies formula (13) is greater than or equal to the minimum confidence, *X*⟶*Y* is a strong association rule [17].

(12) $$\begin{array}{c} Support\left(X⟶Y\right)\geq \mathrm{Min}\_Sup\text{,} \end{array}$$

(13) $$\begin{array}{c} Confisence\left(X⟶Y\right)\geq \mathrm{Min}\_Conf\text{.} \end{array}$$

Join operation: generate itemsets (*k*+1)− by joining two frequent itemsets with the same item (*k* − 1) prefix *k*− for example, there are two 3-itemsets:

(14) $$\begin{array}{c} I_{31}=\left\{A,B,C\right\},\\ I_{32}=\left\{A,B,E\right\}. \end{array}$$

They have the same first two terms {*A*, *B*}, so *I*_31_ and *I*_32_ join to get the 4-term set given as follows:

(15) $$\begin{array}{c} I_{34}=\left\{A,B,C,E\right\}\text{.} \end{array}$$

### 2.3. Algorithm Experiment and Analysis

#### 2.3.1. Experimental Process

According to the two improvement strategies proposed above, corresponding optimization strategies are implemented in the algorithm execution process. The improved BDEclat algorithm is divided into two stages: data pre-processing stage (converting horizontal structure of source data into vertical structure) and the frequent itemset generation stage (iteratively mining all high-order frequent itemsets) [18].

The first stage is the data preprocessing stage, which transforms the horizontal data structure into vertical data structure in the transaction database and forms candidate 1-item set C1. The second stage is the frequent item set mining stage. In this stage, candidate 1-item set C1 after pre-processing is taken as the input, and the iterative calculation of frequent item sets of all items is realized through a double-layer cycle.

The experimental platform is Intel Core I5-3230m processor, 8 GB memory, Windows 7 OPERATING system PC, algorithm implementation platform is Eclipse, and the programming language is Java [19]. Data sets used in the experiment are real and synthetic public test data sets commonly used in association algorithm research. Among them, the Mushroom data set contains different attribute information of various mushrooms. The Chess data set lists the positions of Kings relative to Kings at the end of a Chess game; Data sets T10I4D100K and T40I10D100K were synthesized by the IBM QuestMarket-Basket Synthetic Data Generator of IBM Almaden Quest Research Group [20]. At the same time, the statistical characteristics of the four data sets were compared. The execution of the experiment, in order to ensure the precision of the whole experiment, and reliability of the results, try to eliminate the execution environment change and the background process influence on the conclusion, the deviation of the result is unpredictable. This experiment support each group of data sets of different degrees, respectively recording 10 groups of experimental data, the average correlation analysis, and calculation of the reentry after processing.

#### 2.3.2. Interpretation of Results

Based on the original algorithm Eclat, the algorithm BEclat uses the bit storage mechanism to optimize the array and matrix storage methods, and the memory consumption when compressing data storage; the algorithm DEclat uses deep pruning on the basis of the original algorithm Eclat to reduce irrelevant itemsets in the iterative calculation process, compressing Candidate Item Set Size. The BDEclat algorithm integrates two improved strategies on the basis of the original algorithm Eclat to improve the execution efficiency of the algorithm [21]. By comparing the time consumption and memory consumption of the four algorithms on the four types of data sets, the effectiveness of the improved strategy is verified. The experimental results show the time consumption comparison of BDEclat algorithm on four data sets, as shown in Figures 2–5.

Comparing two sets of algorithms based on BitSet binary storage and Set collection storage BDEclat/DEclat and BEclat/Eclat, the time complexity of the Mushroom Chess T10I4D100K and T40I10D100K data sets decreased by an average of 66.31 times, 84.74 time, 13.37 time, 64.5 times. After multi-angle deep pruning, compared with BDEclat/BEclat and DEcla/Eclat, the time complexity was reduced by 7.73 times, 2.61 times, 4.09 times, and 3.49 times on average under the four data sets.

In order to verify the accuracy of the algorithm, the experiment compares the number of frequent item sets mined by the improved BDEclat algorithm and Eclat algorithm under the different support degree of four different data sets. The experimental results show that the improved algorithm under the different support of four data sets, the number of frequent itemsets mining in complete accord with Eclat algorithm, the accuracy of the algorithm is not reduced because of time and memory consumption and weaken improved algorithm to the data sets of different statistical properties improvement effect is slightly different, its promotion effect is more obvious on the intensive data set. On the premise of ensuring the accuracy of mining results, the algorithm can effectively reduce the time and space consumption, indicating that the improved algorithm has universality and effectiveness, and the research has practical significance and value.

## 3. Empirical Analysis on the Evaluation of Management Status of Listed Enterprises

According to the research purpose of this paper, applying the optimized association rule algorithm, 19 unicorn companies listed in 2021 (see Table 1) are selected as the research samples for the convenience and feasibility of data collection. The business scope covers Internet, automobile, live broadcasting, medicine and other fields, and basically covers the current business field of Chinese unicorn enterprises. It can represent the development status of unicorn enterprises and conform to the research purpose of unicorn enterprise operating efficiency evaluation in this paper.

This paper analyzes the two indexes of asset scale and shareholders' equity (see Table 2). First of all, from the perspective of asset scale, in 2021, the total asset scale of 19 listed unicorns reached 568.351 billion yuan, and the average asset scale was 29.913 billion yuan, which shows that there is a big difference among enterprises. At the same time, only B enterprise, H enterprise, and K enterprise reached the average size, accounting for only 31.58%, and thirteen companies are below average size. Among the 19 enterprises, H enterprise has the largest asset scale, reaching 145.228 billion yuan, while I enterprise has the smallest asset scale, only 102 million yuan, with a difference of more than 140 billion yuan between the maximum and minimum value. Second, from the perspective of shareholder equity, the shareholder equity scale of China's 19 listed unicorns in 2021 is 326.788 billion yuan, with an average size of 17.199 billion yuan, among which only 6 enterprises reach the average. On the whole, large group enterprises such as H and L enterprises have increased the average, and the overall scale of most listed unicorn enterprises is relatively low, among which there are 9 enterprises with assets of less than 10 billion yuan. However, overall, the development scale of unicorn enterprises is still higher than the average asset scale of listed companies nationwide (A-share).

As for income and profit, this paper analyzes the two indexes of operating income and net profit (see Table 3). First of all, in terms of the scale of operating revenue, the total operating revenue of the 19 listed unicorn enterprises will reach 361.987 billion yuan in 2021. The average revenue was 19.052 billion yuan, and four companies reached the average revenue scale, accounting for 21.05%. But it is still nearly 60% higher than the average revenue of 12.543 billion yuan of listed companies nationwide in 2021. The average net profit of 19 companies was −6.826 billion yuan, only 9 enterprises made a profit, and 10 enterprises showed a loss, reflecting that they are still in the growth stage, and profitability is limited. Therefore, on the whole, the profitability of the 19 enterprises is average, and only H enterprise and J enterprise, and other large enterprises are profitable. However, from the perspective of the profit rate, Q enterprise has the highest profit rate, which reaches 69.21%, while L enterprise has the lowest profit rate, which is close to -200%. There are great differences in the growth stages of each enterprise's business field.

### 3.1. Selection of Input-Output Indicators

#### 3.1.1. Input Indicators

1. Total assets: unicorn enterprises are typical scale economy enterprises, and total assets include all assets of the enterprise, which can better reflect the scale of the enterprise. Therefore, the index of total assets is in line with the development characteristics of unicorn enterprises.
2. Operating costs: operating cost is the main input of a company and is directly related to operating revenue, which can be divided into main business costs and other business costs. Considering the difference in the proportion of the main business of different unicorn enterprises, operating cost is selected as the input index.

#### 3.1.2. Output Indicators

Currently, most unicorns have yet to turn a profit. Combined with the principle of nonnegative output index, which output index to choose is very important. Operating income is the most intuitive indicator to reflect the operating results of unicorn enterprises. Therefore, this paper chooses operating income as the output indicator in order to show the value of unicorn enterprises.

#### 3.1.3. Data Description

According to the above input-output indicators, descriptive statistics of the statistical data of 19 listed unicorns listed in 2021 are shown in Table 4.

According to the analysis in Table 4, during the three years from 2019 to 2021, both the input index and output index maintained rapid growth, with the average growth rate of input index reaching 70.68% and 65.58% respectively, and the maximum growth rate of output index reaching 72.07. This is closely related to the development characteristics of unicorns. In terms of standard deviation, operating costs vary the most from company to company.

#### 3.1.4. Correlation Analysis

In this section, SPSS21.0 software is used to verify the correlation of input-output indicators for three years from 2019 to 2021 by non-parametric Kendall's tau_b rank method. The verification results show that *K* values between the input-output indicators are all less than 0.05, passing the significance test, and there is a significant positive correlation. It shows that the two input indicators selected in this paper and one output indicator are reasonable and can better reflect the operating conditions of the sample companies.

### 3.2. Empirical Results and Analysis

Based on the input-output data of 19 listed unicorn enterprises for three consecutive years from 2019 to 2021, this section calculates the pure technical efficiency and then calculates the scale efficiency, so as to evaluate the operating efficiency of enterprises. The data processing software in this paper is MaxDEA. In this section, the data results calculated by MaxDEA software are compared and analyzed from horizontal and vertical dimensions. A more comprehensive analysis compares the relative efficiency, judges the effectiveness of the efficiency, analyzes the causes, and obtains the results.

#### 3.2.1. Lateral Result Analysis

The horizontal analysis in this section is based on the average original data of input and output indicators of 19 listed unicorn enterprises in the three years from 2019 to 2021 to calculate the average operating efficiency of these three years. The calculated results (average technical efficiency value, average pure technical efficiency value, average scale efficiency value, corresponding learning benchmark) are shown in Table 5. Through horizontal analysis, we can understand the overall operating efficiency level of this stage, and preliminarily evaluate the efficiency value of these three years.

According to the calculation results in Table 5, the average technical efficiency of the 19 listed unicorn enterprises is 0.5305, objectively reflecting the low level of overall operating efficiency. Among them, there are only 2 enterprises with technical efficiency value of 1, respectively M enterprise and H enterprise, accounting for 10.53%, indicating that there are relatively few enterprises with technical efficiency. Meanwhile, M enterprise has been referred 18 times, and H enterprise has been referred 15 times. In addition, the remaining 17 enterprises are non-technical effective decision-making units, and their efficiency values are all less than 0.9. Q enterprise has the lowest efficiency value, which is only 0.2191, with a gap of 0.7809 from the maximum value, reflecting the large difference in efficiency values among the 17 enterprises. Only 7 enterprises reach the average technical efficiency value, accounting for 36.84%. In terms of the average pure technical efficiency value and scale efficiency value of the 19 listed unicorn enterprises, they are 0.7311, and 0.7439 respectively. Then, for the 17 enterprises with invalid technology, except for M enterprise and H enterprise with effective technology, there are three situations: one is pure technical inefficiency but scale efficiency (pure technical efficiency is less than 1, scale efficiency is 1); Second, pure technical efficiency but no scale efficiency (pure technical efficiency is 1, scale efficiency is less than 1); Third, pure technical scale is inefficient (pure technical efficiency and scale efficiency are all less than 1). Specifically, among the 17 technologically ineffective enterprises, the pure technical efficiency value of three enterprises, K, I, and S, is 1, which is pure technically effective but ineffective in scale, reflecting that these three enterprises are technically capable. Sufficient, but the scale of operation has not yet reached the optimal state, and it has formed a state where pure technology is effective but scale is invalid, making the overall technical efficiency invalid. This reflects that there are problems in the development of technological production capacity and scale of these 14 enterprises, which need to be analyzed from these two dimensions in order to better improve.

#### 3.2.2. Longitudinal Result Analysis

In order to further analyze the operating efficiency differences of listed unicorn enterprises in each year, the longitudinal analysis in this section is based on the input and output index data of 19 listed unicorn enterprises in each of the three years from 2019 to 2021. Calculate the operating efficiency of each year respectively, and conduct a vertical comparative analysis with time series to supplement the shortcomings of horizontal analysis, so as to achieve the goal of comprehensive analysis of enterprise operating efficiency. During 2019–2021, through the analysis of the efficiency of the three years without a business for three consecutive years, technical efficiency value is 1, continuous efficiency does not implement effective state, for the 19 companies in 2019–2021 of technical efficiency change as shown in Figure 6, you can see three years of technical efficiency change is bigger, only M enterprise for two consecutive years of the state of the efficiency value is 1.

According to the changing chart of technical efficiency in the three years from 2019 to 2021, the trend can be divided into five types by comparing its changing trend. First, the overall trend is increasing year by year, indicating that its technical efficiency is gradually rising, approaching effective and showing a good trend. Second, the overall trend is declining year by year, indicating that the technical efficiency is gradually declining, and the distance from the production frontier is getting further and further, and there may be problems in operation. Third, the overall trend fell first and then increased, indicating that problems were encountered halfway, but have gradually improved; Fourth, the overall trend increases first and then decreases. The efficiency of this type of enterprise is gradually improving in the early stage, but it shows a trend of deterioration in the later stage, and gradually separates from the production frontier, which may have potential problems. Fifth, the overall trend is stable, which has remained stable for three consecutive years without any improvement or decline. According to the same evaluation and analysis method above, the change trend of pure technical efficiency value of 19 companies was analyzed. It can be concluded that among the 19 enterprises, only two enterprises, O and K, saw the changing trend of pure technical efficiency increase year by year, and the proportion was only 10.53. The number of enterprises with the overall trend of decline or increase first and then decline also reached 14, reaching 73.68%, which objectively reflects the relatively low technological production capacity of sample enterprises and the possibility of deterioration. This section selects the sample enterprises studied in this paper, analyzes the operating fundamentals of the sample enterprises, and preliminarily analyzes the basic operating conditions of 19 listed unicorn enterprises. Then, according to the selection principle of the DEA evaluation index, total assets operating cost is selected as the input index and operating income as the output index. CCR and BCC models are selected as evaluation models of the operating efficiency of unicorn enterprises according to the research purpose. Then, relevant data of sample enterprises from 2019 to 2021 are inserted for empirical analysis from horizontal and vertical dimensions. The analysis shows that the operating efficiency gap between 19 unicorn enterprises is large and the efficiency value is low. In the horizontal comparative analysis, only two enterprises have effective technology. In the longitudinal comparison analysis, there are no enterprises with effective technology for three consecutive years, and the main reason for the low-efficiency value of enterprises is that the return to scale is in a decreasing state, indicating that the operation scale is too large, business complexity increases the difficulty of the operation and reduces the operation efficiency.

## 4. Conclusion

On the basis of relevant research abroad, this paper compares and analyzes the advantages and disadvantages of different efficiency evaluation methods, and selects the input-output index of enterprise operating efficiency evaluation based on the association rule algorithm and data set DEA method. Two classical models are determined as the analysis basis, and then the operating efficiency of 19 listed unicorn companies from the horizontal and vertical perspectives is comprehensively evaluated. Conclusions are given as follows.

Lateral analysis conclusion. Through the calculation and analysis of the average operating efficiency of 19 listed unicorn enterprises during the three years from 2019 to 2021, it is found that the average technical efficiency value is 0.5305, objectively reflecting the low level of overall operating efficiency. Among them, only two enterprises, M enterprise and H enterprise, are effective with DEA technology, while 17 enterprises are not effective. In terms of specific reasons, it is directly related to the production scale of technical capacity. In particular, six companies, including Q, O and D, are in the stage of increasing returns to scale, indicating that they need to increase the scale of operations and investment to improve their efficiency and management status; The returns to scale of 11 enterprises, including J Enterprise, B enterprise, and A enterprise, are in A decreasing state, indicating that their business scale is too large and their business scope is wide. It indicates that the complexity of business increases the difficulty of operation, and the vertical analysis results show that the efficiency can be improved only by reducing the scale of operation. Based on the annual calculation and analysis of the operating efficiency of 19 listed companies in the three years from 2019 to 2021, it can be seen from the change trend of pure technical efficiency and scale efficiency of technical efficiency, only two enterprises, O and K, maintain an increasing trend in the efficiency values of the three categories. The three types of efficiency values of D enterprise, Q enterprise, A enterprise, and P enterprise all showed A downward trend, which objectively confirmed that the overall efficiency level of listed unicorn enterprises was low and showed A downward trend, and also reflected the urgency of unicorn enterprises to improve operational efficiency. This also shows that many current unicorns are the one-sided pursuit of business scale, striving for capital market financing, doing high valuation, and going on the pursuit of the purpose of listing. Through the research of this paper, it is found that the average pure technical efficiency of 14 out of 19 companies is less than 1, which objectively reflects that the overall technical capability needs to be improved. Therefore, while promoting the normal operation and development of enterprises, it is necessary to increase investment in RESEARCH and development and cultivate talents with innovative abilities. In particular, the investment in new technology and the development of new products, the innovation of business model, and the improvement of operation and management mode should be emphasized, and the scientific research and innovation ability should be constantly strengthened. The investment in innovation ability should be converted into output as soon as possible, so as to improve the production technology level and enhance the core competitiveness of enterprises.

## Figures and Tables

**Figure 1:** Enterprise operating model.

**Figure 2:** Algorithm on the mushroom time and memory consumption comparison.

**Figure 3:** The algorithm compares time and memory consumption on Chess.

**Figure 4:** Algorithm on T10I4D100K time and memory consumption comparison.

**Figure 5:** Algorithm on T40I10D100K time and memory consumption comparison.

**Figure 6:** Chart of changes in technical efficiency values of 19 listed unicorn companies from 2019 to 2021.

**Table 1:** A brief list of listed unicorn companies.

Serial number	Enterprise abbreviation	Time to market
1	A enterprise	2021.03.28
2	B enterprise	2021.03.29
3	C enterprise	2021.05.04
4	D enterprise	2021.05.11
5	E enterprise	2021.06.11
6	F enterprise	2021.06.27
7	G enterprise	2021.06.29
8	H enterprise	2021.07.09
9	I enterprise	2021.07.12
10	J enterprise	2021.07.13
11	K enterprise	2021.07.26
12	L enterprise	2021.09.12
13	M enterprise	2021.09.14
14	N enterprise	2021.09.20
15	O enterprise	2021.09.28
16	P enterprise	2021.11.26
17	Q enterprise	2021.11.27
18	R enterprise	2021.12.06
19	S enterprise	2021.12.12

**Table 2:** Development scale of 19 listed unicorn enterprises in 2021 (unit: RMB 100 million).

Serial number	Enterprise abbreviation	Asset size	Stockholders' equity
1	A enterprise	117.90	71.91
2	B enterprise	452.60	181.56
3	C enterprise	134.74	102.67
4	D enterprise	82.06	56.45
5	E enterprise	742.84	349.38
6	F enterprise	76.29	23.72
7	G enterprise	38.04	28.29
8	H enterprise	1471.28	733.23
9	I enterprise	1.32	0.55
10	J enterprise	78.34	35.46
11	K enterprise	428.82	192.23
12	L enterprise	191.43	81.50
13	M enterprise	24.52	16.08
14	N enterprise	1214.62	845.10
15	O enterprise	8.02	5.21
16	P enterprise	167.91	105.27
17	Q enterprise	37.54	31.06
18	R enterprise	42.59	38.61
19	S enterprise	487.64	364.59
Average value		305.18	171.73
Total value		5798.5	3262.87

**Table 3:** Annual revenue and profit status of 19 listed unicorn enterprises in 2021 (unit: RMB 100 million).

Serial number	Enterprise	Operating receipt	Retained profits	Profit margin (%)
1	A enterprise	41.29	−5.65	−13.68
2	B enterprise	249.89	−90.61	−36.26
3	C enterprise	33.38	−9.12	−27.32
4	D enterprise	46.63	−19.38	−41.56
5	E enterprise	296.11	33.87	11.44
6	F enterprise	33.15	−15.38	−46.40
7	G enterprise	12.25	0.08	0.65
8	H enterprise	1749.15	135.54	7.75
9	I enterprise	0.63	0.018	2.86
10	J enterprise	28.12	21.62	76.88
11	K enterprise	131.2	−102.17	−77.87
12	L enterprise	49.51	−96.39	−194.69
13	M enterprise	28.14	−19.46	−69.15
14	N enterprise	652.27	−1154.77	−177.04
15	O enterprise	9.112	0.748	8.21
16	P enterprise	52.56	5.30	10.08
17	Q enterprise	7.6	5.26	69.21
18	R enterprise	9.03	−4.86	−53.82
19	S enterprise	189.85	18.32	9.65
Average value		190.52	−68.26	−35.83
Total value		3619.87	−1297.03	−35.83

**Table 4:** Descriptive statistics of input-output variables of sample unicorn enterprises (unit: RMB 100 million).

2019	Total assets	Operating costs	Operating receipt
Maximum value	517.17	671.85	684.34
Minimum value	0.3	0.07	0.58
Mean value	102.68	67.55	64.35
Standard deviation	2.12	2.08	1.86
2020	Total assets	Operating costs	Operating receipt
Maximum value	898.7	1090.13	1146.25
Minimum value	0.65	0.64	0.61
Mean value	173.23	109.57	115.63
Standard deviation	1.91	1.98	1.74
2021	Total assets	Operating costs	Operating receipt
Maximum value	1452.28	1787.28	1749.15
Minimum value	1.02	0.98	0.63
Mean value	299.13	185.20	190.52
Standard deviation	1.73	1.99	1.76
Mean value of 3 years	Total assets	Operating costs	Operating receipt
Maximum value	952.88	1183.09	1193.25
Minimum value	0.66	0.74	0.61
Mean value	191.68	120.77	123.50
Standard deviation	1.75	1.91	1.70

*Note.* In view of the large gap between the input-output variables of various enterprises, the natural logarithm is adopted to calculate the standard deviation.

**Table 5:** Average efficiency distribution table of 19 listed unicorn companies in 2019–2021.

No.	DMU	TE	PTE	Se	RTS
1	J enterprise	0.27892	0.47895	0.582356	Decreasing
2	B enterprise	0.58062	0.812606	0.71452	Decreasing
3	Q enterprise	0.21906	0.239146	0.916048	Increasing
4	A enterprise	0.50595	0.656494	0.770696	Decreasing
5	O enterprise	0.81039	0.916603	0.884126	Increasing
6	D enterprise	0.76488	0.76588	0.998694	Increasing
7	N enterprise	0.39471	0.747379	0.528137	Decreasing
8	R enterprise	0.49139	0.522304	0.940815	Increasing
9	E enterprise	0.39464	0.978665	0.403244	Decreasing
10	K enterprise	0.63365	1	0.633659	Decreasing
11	C enterprise	0.23624	0.282091	0.837472	Decreasing
12	I enterprise	0.75923	1	0.759236	Increasing
13	M enterprise	1	1	1	Constant
14	S enterprise	0.33389	1	0.333891	Decreasing
15	P enterprise	0.41269	0.572373	0.721021	Decreasing
16	L enterprise	0.37805	0.636159	0.594272	Decreasing
17	H enterprise	1	1	1	Constant
18	F enterprise	0.43646	0.828941	0.526537	Decreasing
19	G enterprise	0.447786	0.452577	0.989411	Increasing
Average mean		0.53045	0.7310614	0.743902	

## Data Availability

The data used to support the findings of this study are available from the corresponding author upon request.
